The article "Therapeutic Effects and Metabolic Spectrum of Traditional Chinese Medicine Hengqing II Prescription on Alzheimer's Disease" was published in 2022. Journal: Evid Based Complement Alternat Med.

# Therapeutic Effects and Metabolic Spectrum of Traditional Chinese Medicine Hengqing II Prescription on Alzheimer's Disease

**DOI:** 10.1155/2022/5912396

**Published:** 2022-08-02

**Authors:** Shengxi Meng, Shaopeng Li, Huize Chen, Chujun Deng, Zeyu Meng, Yimo Wang

**Affiliations:** ^1^Department of Traditional Chinese Medicine, Shanghai Jiao Tong University Affiliated Sixth People's Hospital, Shanghai 200233, China; ^2^Shanghai Sensichip Infotech, Shanghai 200331, China; ^3^The Second Clinical Medical College, Heilongjiang University of Chinese Medicine, Harbin 150040, China

## Abstract

Alzheimer's disease (AD) seriously damages elders' social and daily abilities around the world. Traditional Chinese medicine (TCM), a rich drug resource bank, could help research AD. In order to explore the role of TCM in AD treatment, 86 AD patients were recruited from the hospital, then treated with Hengqing II prescription and donepezil hydrochloride. The cognitive and serum lipid levels were investigated before and after treatment. The patient's urine was collected after three months of treatment. Metabolites in the urine samples were extracted with methanol and detected on the UHPLC-MS platform. Results proved that Hengqing II can improve cognitive levels and reduce the levels of Hcy, D-D, FIB, Apo B, TC, and LDL-C compared with donepezil hydrochloride (*P* < 0.05). The results of multivariate statistical analysis revealed that the metabolism of HQII was significantly different compared with Control groups. A total of 66 differential metabolites were found in this comparison (50 were down-regulated and 16 were up-regulated). Four amino acid pathways and one linoleic acid pathway were found through these metabolites. After receiver operating characteristic analysis, it was suggested that palmitic acid, palmitoleic acid, linoleic acid, oleic acid, SAH, and methionine can be used as biomarkers for treating AD, while the effects of daidzein, genistein, and naringenin on the treatment of AD need to be further studied.

## 1. Introduction

Alzheimer's disease (AD) is a degenerative disease in the central nervous system and is mainly characterized by cognitive decline [1–3]. It has become a major public concern due to symptoms of AD being difficult to diagnose at the early stage [4]. It is estimated that by 2050, the number of patients with AD in the world will exceed 130 million [5]. Thus, it is urgent to strengthen the research on the diagnosis and treatment of AD. However, the pathogenesis of AD is not fully explained and the development of drugs for treating AD is still full of challenges. At present, the discovery of new biomarkers is of great help in the treatment of AD. Thus, many researchers and resources are invested in the research on biomarkers of AD every year [6–8]. We noticed that numerous studies focus on biomarkers of AD patients' blood and brain, while there are relatively few studies researching biomarkers related to AD patients' urine [9, 10]. The changes in metabolites in the urine of AD patients aroused our interest. Whether new biomarkers can be found in AD patients' urine and whether there are significant differences between metabolites in urine and metabolites in blood and brain need to be confirmed.

The article "Therapeutic Effects and Metabolic Spectrum of Traditional Chinese Medicine Hengqing II Prescription on Alzheimer's Disease" was published in 2022. Journal: Evid Based Complement Alternat Med.

Traditional Chinese medicine (TCM) is one of the most influential alternative medicines in the world. Faced with the challenges of treating AD, TCM has gained importance in the prevention and treatment of AD, with a bright future [11–14]. To date, there is no theoretical basis for using TCM prescription to treat AD. According to our clinical practice, TCM Hengqing II prescription has satisfactory effects on the treatment of AD. However, due to many plant components and complex chemical composition in Hengqing II, we do not know, which component plays a major role in the treatment of AD. Meanwhile, as a common method for diagnosing AD, scale tests will be affected by the subjective of AD patients, thus resulting in inaccurate data. Therefore, studying the metabolic changes of AD patients after taking Hengqing II can help clarify the main components of Hengqing II and provide objective evidence for the diagnosis of AD as well. To date, metabolite detection has become more efficient and reliable [15, 16], and it is a powerful approach for studying AD pathogenic processes and biomarkers. Therefore, to gain a deeper understanding of AD pathology and provide a data basis for TCM diagnosis of AD, in this study, the effects of Hengqing II on the metabolic spectrum were explored by UHPLC-MS, and reliable biomarkers were discovered.

## 2. Materials and Methods

### 2.1. Recruitment and Grouping of AD Patients and Urine Collection

From December 2016 to December 2018, 86 patients suffering from AD were treated in the Shanghai Jiao Tong University Affiliated Sixth People's Hospital, and they were recruited as the research population. This study was approved by the hospital ethics committee (Approval No. 2019–12). The AD patients had obvious mental symptoms and cognitive impairment and met the diagnostic criteria of AD in the *Chinese Classification and Diagnostic Criteria of Mental Disorders (3rd Edition)*. According to TCM syndrome differentiation, 58 patients were in the KDPS group and 28 patients were in the non-KDPS group. Urine samples were collected to detect metabolic differences between the two groups. After that, the KDPS group was equally divided into two groups by the random number table method. One group took Hengqing II formula once a day, no more than five times a week (HQII group), and another group took donepezil hydrochloride tablets (5 mg/tablet) simultaneously (Control group). Hengqing II consists of 11 kinds of TCM (Table 1). The herbs were extracted using boiling water for 2 h. The extract was filtered, evaporated on a rotary vacuum evaporator, and lyophilized using a freeze-dryer. Most AD patients recruited were accompanied by other diseases such as hypertension and diabetes. Therefore, in order to eliminate such interference in the treatment process, relevant patients were provided corresponding drug treatment. Urine samples were collected from the HQII group and Control group after three-month treatment. Before detection, urine samples were stored in an environment of minus 80°C.

The article "Therapeutic Effects and Metabolic Spectrum of Traditional Chinese Medicine Hengqing II Prescription on Alzheimer's Disease" was published in 2022. Journal: Evid Based Complement Alternat Med.

### 2.2. Scale Tests of AD Patients Taking Hengqing II and Control Group

The scale tests of AD patients after taking Hengqing II and donepezil hydrochloride tablets were measured before therapy, 1 month, and 3 months of therapy. Montreal Cognitive Assessment (MoCA) was used to evaluate the cognitive impairment of patients. The scale has 30 points. If the score is higher, the mental state will be better. The cognitive function of patients was evaluated by Alzheimer's Disease Assessment Scale-Cognitive Subscale (ADAS-Cog), with a score range of 0–75 points. If the ADAS-Cog score is higher, the cognitive ability of patients will be worse. The Activities of Daily Living (ADL) scale was used to evaluate the ability of daily living of patients. The score range was 14–64 points. If the ADL score is higher, the patients' ability of daily living will be worse. The Personal and Social Performance (PSP) scale was used to evaluate the behavior ability of patients. 71–100 points represent slight difficulty, 31–70 points indicate ability defect, and 0–30 points denote low function and need support or monitoring. Cohen Mansfield Aging Inventory (CMAI) was used to evaluate the frequency of patients' aggressive behavior. If the CMAI score is higher, the behavior will be more aggressive.

### 2.3. Detection of Serum Biochemical Indexes in AD Patients Taking Hengqing II Formula and Control Group

Venous blood (8 mL) was taken from HQII and Control groups (fasting 12 h) before therapy, 1 month, and 3 months of therapy, and serum was separated. The contents of homocysteine (Hcy), apolipoprotein A1 (Apo A1), apolipoprotein B (Apo B), total cholesterol (TC), low-density lipoprotein cholesterol (LDL-C), and high-density lipoprotein cholesterol (HDL-C) were measured by HITACHI7600 automatic biochemical analyzer. The levels of plasma D-D and fibrinogen (FIB) were detected by the turbidimetric inhibition immune method with SYSMEX CS5100 System.

The article "Therapeutic Effects and Metabolic Spectrum of Traditional Chinese Medicine Hengqing II Prescription on Alzheimer's Disease" was published in 2022. Journal: Evid Based Complement Alternat Med.

### 2.4. Metabolites Were Extracted from Urine Samples

The samples were thawed slowly on ice. After that, 100 *μ*L urine per sample was transferred into a 1.5 ml centrifuge tube and 300 *μ*L extract (pure methanol) was added. With vortex for 30 s and ultrasonic treatment at 4°C for 30 min, the centrifuge tubes stood at −20°C for 1 hour and centrifuged at 15000 rpm for 10 min. Subsequently, 200 *μ*L supernatant was transferred into the injection vial and a 5 *μ*L internal standard (1 mg/ml 2-chlorophenylalanine) was added for UHPLC-MS detection. The supernatant was mixed in all tubes and took 500 *μ*L and 12.5 *μ*L internal standards were used as quality control (QC) samples. All samples were stored in an environment of 4°C for no more than 12 h waiting for on-board detection.

### 2.5. Operating Parameters of Ultra-High Performance Liquid Chromatograph-Mass Spectrometer

Ultra-high performance liquid chromatography (AB SCIEX LC-30A) equipped with an XBridge amide column (4.6 mm × 250 mm, 3.5 *μ*m) was used to separate materials in urine, and the injection volume was 4 *μ*L. The composition of liquid phase A was pure water, with 10 mM ammonium formate and 0.1% (v/v) formic acid. Liquid phase B is chromatographic grade acetonitrile. During elution, the flow rate of the mobile phase was 0.8 mL/min and the column temperature was 40°C. The gradient changes of mobile phase B were 95% (0.5 minutes), 95%–65% (0.5–10 minutes), 65%–40% (10–14 minutes), 40% (14–16 minutes), 40%–95% (16–16.1 minutes), and 95% (16.1–20 minutes). The mass spectrometer (AB SCIEX TripleTOF5600+) equipped with electron spray ionization (ESI) was used to ionize molecules. The voltage of ESI was 4200 V and the temperature was 350°C. Nitrogen was used as sheath gas and auxiliary gas of ESI, and the flow rates were 35 Arb and 15 Arb, respectively. All data were collected using a data-dependent acquisition (DDA) model with m/z ranging from 100 to 1000. The isolation span was 3 Da and the activation time was 30 ms. The high-resolution Fourier transform approach was used. MS1's resolution was 60000, whereas MS2's resolution was 15000.

### 2.6. UHPLC-MS Results Processing

The format obtained from the UHPLC-MS platform was a raw data file. The file was converted to ABF format and MS-DIAL software was used to extract peaks, contrast peaks, filter peaks, fill gaps, and identify materials. The mass threshold of peak extraction was 5 ppm, the retention time threshold was 0.2 min, and the signal-to-noise ratio threshold was 3. The compounds were identified using a data-dependent acquisition pattern with 60 matching factor score thresholds. After processing, a table containing metabolite name, molecular weight, m/z, retention time, and peak area was obtained. According to the material information on the PubChem and Human Metabolome Database (HMDB) websites, another manual identification was conducted to ensure reliable metabolites. PCA, OPLS-DA analysis, and permutation tests were performed on the peak area using SMICA-P 14.0 software to analyze the metabolic differences between the two groups [17]. PCA projects multidimensional data to two or three dimensions through variance, so that it can quickly observe whether there are differences between groups [18, 19]. Compared with PCA, OPLS-DA includes orthogonal conversion, which filters out the data irrelevant to the model classification [20]. A *p*-value less than 0.05 and a VIP value greater than 1 were used as the conditions for screening differential metabolites. Metaboanalyst website was used for pathway analysis and ROC analysis, and SPSS 13.0 statistical software was the tool for data processing.

The article "Therapeutic Effects and Metabolic Spectrum of Traditional Chinese Medicine Hengqing II Prescription on Alzheimer's Disease" was published in 2022. Journal: Evid Based Complement Alternat Med.

## 3. Results

### 3.1. Effects of Taking Hengqing II on the Scale Tests of AD Patients

After taking Hengqing II and donepezil hydrochloride tablets, the MoCA and PSP scores of the HQII group after 3 months improved more significantly than those of the Control group after 3 months. The ADAS-Cog, ADL, and CMAI scores of the HQII group after 3 months were obviously lower than those of the Control group after 3 months (Table 2), which showed that Hengqing II was better than donepezil hydrochloride in treating AD after taking at the same time.

### 3.2. Effects of Taking Hengqing II on Serum Biochemical Indexes in AD Patients

After treatment with Hengqing II and donepezil hydrochloride, the contents of Hcy, D-D, FIB, Apo B, TC, and LDL-C in the HQII group after 3 months were lower than in the Control group after 3 months of treatment. The levels of Apo A1 and HDL-C in the HQII group after 3 months of treatment were significantly higher than those in the Control group (Table 3). These results revealed that Hengqing II can reduce the levels of Hcy, D-D, FIB, Apo B, TC, and LDL-C in AD patients and the effects were better than donepezil hydrochloride tablets. Combined with the previous results of Hengqing II in improving the cognitive ability of AD patients, it was speculated that the Hengqing II formula can regulate the metabolites of AD patients, especially lipids. Therefore, a follow-up metabolomics difference study was conducted.

### 3.3. PCA and OPLS-DA Analysis of Metabolites' Data

It can be observed that the KDPS group was significantly different from the non-KDPS group, and the HQII group was significantly different from the Control group (Figures 1(a) and 1(b)). In Figures 1(c) and 1(d), the HQII and KDPS samples could be distinguished from the Control and non-KDPS individuals. It was also found that the separation effects of KDPS on non-KDPS are not as good as that of the HQII group and Control group in the center of a confidence interval, which showed the metabolic differences between HQII and Control groups were greater than the previous comparison. In permutation test plots (Figures 1(e) and 1(f)), the OPLS-DA models exhibited a well fit, which demonstrated that the urine metabolomics signature differs between the two groups. These metabolomics profiles of KDPS and non-KDPS suggested that AD categorization based on TCM syndrome distinction was dependable and practicable. The significant differences between the HQII group and Control group also confirmed the effective impacts of HQII on the scale tests and serum indicators. Subsequently, we focused on analyzing the effects of Hengqing II on urine metabolites in AD patients.

The article "Therapeutic Effects and Metabolic Spectrum of Traditional Chinese Medicine Hengqing II Prescription on Alzheimer's Disease" was published in 2022. Journal: Evid Based Complement Alternat Med.

### 3.4. Differential Metabolites between the HQII and Control Group

After observing significant differences in metabolic profiles between the HQII group and the Control group, all metabolites found were screened. The *p* value of the student's test and VIP value in OPLS-DA analysis were used as screening conditions. VIP is variably important in the projection. If the VIP value is greater, the contribution of the variable to the differences between the two groups will be greater. When the *p* value was less than 0.05 and VIP was greater than 1, there were 66 differential metabolites in the HQII group compared with the Control group (Table 4). Among these different substances, amino acids, long-chain fatty acids, aromatic compounds, purine derivatives, sugar derivatives, pyrimidine derivatives, and small molecular organic acids were found. In addition, three flavonoids appeared in differential metabolites. Flavonoids may come from plant components in the Hengqing II prescription, which requires our in-depth analysis.

Heatmap was used to visualize the relative contents of metabolites in urine samples (Figure 2). It can be clearly observed that a large number of metabolites in the HQII group (left side of the figure) showed blue down-regulation compared with the Control group (right side of the figure). That meant that the relative contents of almost differential materials of AD patients can be reversed after taking Hengqing II. In order to understand the change range of metabolites more intuitively, variance analysis on these metabolites was conducted, which showed that the Hengqing II treatment significantly reversed the relative abundance of 50 urinary metabolites (Figure 3). It was that Hengqing II prescription may regulate AD by a variety of metabolites. The results of the heatmap and histogram could explain the enhancement of cognitive capacities in AD patients after treatment.

The article "Therapeutic Effects and Metabolic Spectrum of Traditional Chinese Medicine Hengqing II Prescription on Alzheimer's Disease" was published in 2022. Journal: Evid Based Complement Alternat Med.

### 3.5. ROC Analysis of Differential Metabolites

To determine whether these differential metabolites can be used as biomarkers for Hengqing II against AD and to exclude false-positive results, ROC analysis (receiver operating characteristic curve) on differential metabolites were performed. In ROC analysis, AUC (area under curve) value was used as a standard to measure the reliability of metabolites. AUC equals 1, which indicates that the prediction is perfect, AUC between 0.85 and 0.95 implies that the prediction effect is very well, 0.7–0.85 means that the prediction effect is general, 0.5–0.7 refers to a poor effect, 0.5 stands for that the model is meaningless, and less than 0.5 indicates that the prediction is worse than random. Among the differential metabolites we found, palmitic acid had the highest AUC value, and the AUC values of 14 differential metabolites were between 0.85 and 1. 44 differential metabolites ranged from 0.7 to 0.85, and the AUC values of 7 metabolites ranged from 0.65 to 0.7 (Table 4 and Figure 4). It was also noted that the AUC values of fatty acids were generally high and they may be biomarkers.

### 3.6. Pathway Analysis of Differential Metabolites

In order to analyze the relationship between these differential metabolites and the physiological processes, Metaboanalyst 5.0 website was used to locate these differential metabolites on the metabolic pathway. In the HQII and Control groups, the pathways for linoleic acid metabolism, arginine biosynthesis, alanine, aspartate, glutamate metabolism, D-glutamine and D-glutamate metabolism, glycine, serine, and threonine metabolism were discovered (Figure 5).

## 4. Discussion

Firstly, according to the obvious differences in metabolic profile between KDPS and non-KDPS group, it is feasible and meaningful to classify AD through KDPS. At present, there are few studies on the TCM syndrome differentiation of dementia. Liu studied the clinical manifestation of Kangxin capsule in the therapy of senile vascular dementia with kidney deficiency and blood stasis in 2007 [21]. Tan revealed the therapeutic biomarkers of processed *Aconitum Carmichaeli Debx* in treating hydrocortisone-induced Kidney-Yang deficiency syndrome rats [22]. As we all know, this paper was a study on the TCM classification of AD. These results of the multivariate statistical analysis provided a data basis for the therapy of AD by TCM. However, this study did not analyze the changes in metabolites in AD patients after TCM typing, which is worthy of further research.

The article "Therapeutic Effects and Metabolic Spectrum of Traditional Chinese Medicine Hengqing II Prescription on Alzheimer's Disease" was published in 2022. Journal: Evid Based Complement Alternat Med.

In the analysis of the Hengqing II group and the Control group, it was found that Hengqing II significantly improved the clinical manifestation of patients. All indexes in the scale tests have been improved. Meanwhile, Hengqing II also decreased the contents of Hcy, D-D, FIB, Apo B, TC, and LDL-C in serum, which showed the importance of lipid changes in the pathogenesis of AD. According to the papers consulted, fatty acids play a complex role in the pathogenesis of AD, and they are closely related to intestinal microbiota and neuroinflammatory response [23]. In the metabolite analysis, palmitic acid, palmitoleic acid, oleic acid, and linoleic acid were significantly down-regulated and their VIP value was higher than other metabolites, which indicated that they contributed more differences. In the analysis of the metabolic pathway, the linoleic acid metabolism pathway was found and the impact value was much higher than other pathways. In ROC analysis, the AUC values of palmitic acid, palmitoleic acid, linoleic acid, and oleic acid performed very well. The AUC of palmitic acid even reached a maximum. Thus, palmitic acid, palmitoleic acid, linoleic acid, and oleic acid are regarded as biomarkers for curing AD. Many studies on the correlation between fatty acids and AD also accord with the abovementioned views. Palmitic acid can induce neuroinflammatory, and result in neuronal damage [24–26]. However, as an unsaturated fatty acid, linoleic acid has a different performance from palmitic acid in the nervous system. Linoleic acid has protective effects on oxidative stress, neuroinflammation, and memory damage [27, 28]. The significant down-regulation of linoleic acid and palmitic acid in this study may be closely related to the taking of Hengqing II. Therefore, we believe that fatty acids are of great significance in the pathogenesis of AD.

Many amino acids and their derivatives in the screening of differential metabolites and four amino acid metabolic pathways were also found. These results confirmed that amino acids and their derivatives have a great impact on the pathology of AD patients. There are many studies on the effects of branched-chain amino acids (BCAA) on AD, and there is a certain correlation with lipids [29, 30]. In our study, leucine was also remarkably down-regulated, which was consistent with the abovementioned studies. Unfortunately, the AUC value of leucine was not enough. In addition, it was also found that SAH (S-Adenosyl-L-homocysteine) and methionine were significantly down-regulated after treatment, which was highly correlated with AD [31–33]. We also noted that the amino acid with the highest AUC was the dimer of alanine. Lin held the view that higher D-alanine levels are associated with more behavioral symptoms of AD [34]. Combined with ROC analysis, it was suggested that methionine and SAH can be used as biomarkers for treating AD.

The article "Therapeutic Effects and Metabolic Spectrum of Traditional Chinese Medicine Hengqing II Prescription on Alzheimer's Disease" was published in 2022. Journal: Evid Based Complement Alternat Med.

Three kinds of flavonoids were found in differential metabolites, and they are likely to come from a plant component in Hengqing II. It is well known that flavonoids can resist oxidation and improve cell activity. Many studies have proved that flavonoids have antioxidant and anti-inflammatory effects on AD [35–37]. After taking Hengqing II, the relative contents of daidzein, genistein, and naringenin increased significantly, which may help patients reverse the pathology of AD. Ko confirmed that 6,7,4′-Trihydroxyisoflavone (a major metabolite of daidzein) could enhance learning and memory by the cholinergic system and activate the p-CREB/BDNF signaling pathway in mice [38]. Daidzein can also promote hippocampal neurogenesis in middle-aged mice [39]. On the other hand, genistein can alleviate cognitive impairment and correct the behavior of rats by exerting antioxidant and anti-inflammatory effects [40, 41]. Similarly, naringenin can improve the learning and memory ability of AD rats [42, 43]. However, since the AUC value of naringenin was between 0.5 and 0.7, the reliability of the prediction was low. The AUC values of daidzein and genistein were between 0.7 and 0.8, which are general for the prediction. Therefore, whether daidzein, genistein, and naringenin can be used as biomarkers for treating AD, still needs more in-depth and detailed studies. In a word, after taking Hengqing II, the anti-inflammatory and anti-oxidation effects of flavonoids alleviate neuron damage, thus improving the cognitive ability of AD patients. With the recovery of cognitive function, the content of AD biomarkers (palmitic acid, methionine, and SAH) decreased. Of course, these explanations still require more experimental data to confirm.

## 5. Conclusion

The metabolic profiles of HQII and Control groups differed considerably. 66 distinct metabolites were discovered (50 were down-regulated and 16 were up-regulated). After being treated with Hengqing II prescription, some amino and fatty acids were decreased significantly. Three kinds of flavonoids were significantly up-regulated. After ROC analysis, palmitic acid, palmitoleic acid, linoleic acid, oleic acid, methionine, and SAH can be used as biomarkers for treating AD by Hengqing II. These metabolites are conducive for us to understand the disease process of AD and pave the way to successfully treating the condition.

The article "Therapeutic Effects and Metabolic Spectrum of Traditional Chinese Medicine Hengqing II Prescription on Alzheimer's Disease" was published in 2022. Journal: Evid Based Complement Alternat Med.

## Figures and Tables

**Figure 1:** In PCA (a, b) and OPLS-DA analysis (c, d), the sample clustering of the KDPS group and HQII group are significantly different from that of the non-KDPS group and Control group. Grey circles indicate 95% confidence intervals. (e, f) OPLS-DA permutation test plots, indicating that the OPLS-DA model performs very well.

**Figure 2:** The heatmap visualization of protective effects of HQII for AD. The degree of change is marked with different colors, red indicates up-regulation and blue refers to down-regulation. Each row denotes a metabolite, and each column stands for an individual sample.

**Figure 3:** The changes in the relative intensity of target metabolites. Statistical significance was performed using a one-way analysis of variance. A total of 50 metabolites were significantly reversed by HQII treatment. All data are expressed as Mean ± SD.

**Figure 4:** The ROC analysis of palmitic acid, palmitoleic acid, and linoleic acid. The AUC was the area of the shaded part. The horizontal axis is the false-positive probability, and the vertical axis is the true positive probability.

**Figure 5:** The metabolic pathways found according to the differential metabolites. A bubble represents a metabolic pathway. The metabolic pathways with the top five impact values show the pathway names.

**Table 1:** The component content and source of Hengqing II prescription.

TCM name	Amount (*g*)	Source
Yizhiren	30	Fruit of *Alpinia oxyphylla* miq
Huangqi	15	Dry root of *Astragalus membranaceus* (fisch.) bge
Tusizi	10	Mature seed of *Cuscuta chinensis* lam
Chuanxiong	10	Dry stem and root of *Ligusticum chuanxiong* hort
Shudihuang	15	Root tuber of *Rehjnannia glutinosa* libosch
Sangjisheng	10	Dry stem of *Taxillus chinensis* (DC.) danse
Duanshijueming	10	Shell of *Haliotis diversicolor* reeve
Duzhong	10	Dry bark of *Eucommia ulmoides* oliv
Dilong	10	*Pheretima aspergillum* (E. Perrier)
Tianma	10	Stem tuber of *Gastrodia elata* bl
Gouteng	10	Dry stem of *Uncaria macrophylla* wall

**Table 2:** The comparison of scale tests before and 1 month and 3 months after HQII and donepezil hydrochloride treatment in AD patients.

Scale tests	Control group			HQII group		
	Before treatment	1 month after treatment	3 months after treatment	Before treatment	1 month after treatment	3 months after treatment
MoCA score	17.26 ± 2.16	19.11 ± 2.22	23.57 ± 3.03	16.72 ± 4.21	22.58 ± 5.37	26.14 ± 2.10^*∗*^
ADAS-Cog score	34.8 ± 4.7	31.0 ± 3.5	29.6 ± 4.3	34.3 ± 3.6	29.1 ± 3.2	25.2 ± 3.1^*∗*^
ADL score	41.5 ± 5.6	37.2 ± 2.5	35.7 ± 3.7	40.2 ± 4.3	35.5 ± 3.7	29.5 ± 3.4^*∗*^
PSP score	45.63 ± 5.97	51.21 ± 14.37	67.84 ± 14.75	45.74 ± 6.15	59.44 ± 15.88	81.45 ± 16.62^*∗*^
CMAI score	46.92 ± 8.49	41.37 ± 7.62	37.23 ± 6.38	47.89 ± 8.67	38.22 ± 7.21	30.45 ± 6.34^*∗*^

^*∗*^Compared with the Control group after 3 months of treatment, *P* < 0.05.

The article "Therapeutic Effects and Metabolic Spectrum of Traditional Chinese Medicine Hengqing II Prescription on Alzheimer's Disease" was published in 2022. Journal: Evid Based Complement Alternat Med.

**Table 3:** The comparison of serum biochemical indexes before and 1 month and 3 months after HQII and donepezil hydrochloride treatment in AD.

Serum biochemical indexes	Control group			HQII group		
	Before treatment	1 month after treatment	3 months after treatment	Before treatment	1 month after treatment	3 months after treatment
Hcy (*μ*mol/L)	18.37 ± 9.42	18.33 ± 8.79	18.27 ± 8.32	19.22 ± 8.70	17.05 ± 6.13	15.13 ± 5.24^*∗*^
D-D (mg/L)	1.22 ± 0.45	1.21 ± 0.42	1.20 ± 0.48	1.21 ± 0.53	1.16 ± 0.36	1.10 ± 0.26^*∗*^
FIB (g/L)	4.33 ± 2.01	4.12 ± 1.01	4.07 ± 1.02	4.28 ± 1.58	3.35 ± 1.11	2.82 ± 0.95^*∗*^
Apo A1 (g/L)	1.19 ± 0.15	1.20 ± 0.16	1.22 ± 0.15	1.20 ± 0.14	1.38 ± 0.18	1.58 ± 0.21^*∗*^
Apo B (g/L)	0.78 ± 0.09	0.76 ± 0.11	0.75 ± 0.10	0.79 ± 0.07	0.72 ± 0.06	0.68 ± 0.05^*∗*^
TC (mmol/L)	5.01 ± 0.76	4.92 ± 0.62	4.88 ± 0.70	5.02 ± 0.76	4.32 ± 0.62	3.97 ± 0.70^*∗*^
LDL-C (mmol/L)	2.96 ± 0.39	2.95 ± 0.33	2.93 ± 0.35	2.95 ± 0.35	2.52 ± 0.27	2.03 ± 0.28^*∗*^
HDL-C (mmol/L)	0.91 ± 0.11	0.93 ± 0.14	0.94 ± 0.13	0.90 ± 0.10	1.12 ± 0.13	1.19 ± 0.18^*∗*^

^*∗*^Compared with the Control group after 3 months of treatment, *P* < 0.05.

**Table 4:** The differential metabolites between HQII group and Control group.

Name	m/z^1^	RT^2^ (min)	VIP	*p* value	LogFC^3^	AUC^4^
3-Phenyllactic acid	165.06	5.21	1.56	2.48E-02	−4.29	0.777
Palmitic acid	255.23	5.51	2.59	1.10E-12	−3.99	1.000
Stearic acid	283.26	2.66	1.62	2.31E-04	−3.50	0.759
Palmitoleic acid	253.21	2.38	2.02	2.91E-07	−3.39	0.982
Deoxycholate	391.28	7.82	1.21	2.55E-02	−3.23	0.835
Naringenin	271.06	7.59	1.38	2.69E-02	2.99	0.697
Linoleic acid	279.23	2.38	2.19	3.01E-06	−2.54	0.963
Daidzein	253.05	8.81	1.61	9.13E-04	2.51	0.795
Maltitol	343.12	12.51	1.55	1.22E-02	−2.29	0.827
2-isopropylmalic acid	175.06	10.09	1.91	7.79E-05	−2.17	0.879
Oleic acid	281.25	2.47	1.95	1.86E-06	−2.00	0.926
Pyridoxine	168.07	5.49	2.03	3.05E-05	−1.99	0.896
Azelaic acid	187.10	4.20	1.88	1.59E-04	−1.87	0.841
Ala-Ala	159.08	12.17	2.35	5.21E-07	−1.72	0.958
Genistein	269.04	7.85	1.06	2.36E-02	1.71	0.719
Pimelic acid	159.07	10.52	1.72	1.49E-03	−1.71	0.846
L-Cystine	239.02	14.28	1.65	2.01E-03	−1.65	0.815
4-hydroxybenzoic acid	137.02	6.98	1.92	1.42E-07	−1.61	0.875
Phenylacetylglycine	192.07	6.57	1.59	1.85E-03	−1.53	0.796
Citrulline	174.09	12.40	1.08	3.26E-02	−1.52	0.699
3-oxyanthranilic acid	152.03	3.28	1.69	1.18E-05	1.50	0.774
Lactulose	341.11	11.72	1.65	1.77E-02	−1.50	0.847
Taurocholic acid	514.28	7.21	1.55	4.97E-06	1.49	0.875
Hypoxanthine	135.03	6.86	1.98	1.38E-05	1.47	0.890
DHEA sulfate	367.16	2.07	1.93	2.94E-05	1.47	0.839
Allantoin	157.04	7.46	1.89	8.08E-05	−1.41	0.833
Indolelactic acid	204.07	5.72	1.36	2.25E-02	−1.38	0.743
3-hydroxybenzaldehyde	121.03	5.56	1.38	3.31E-04	−1.30	0.761
Threonic acid	135.03	10.99	1.31	1.28E-03	−1.30	0.755
L-homocarnosine	239.11	12.88	1.04	6.95E-03	−1.30	0.670
3′-AMP	346.04	6.04	1.90	1.08E-06	−1.26	0.917
N2-acetylornithine	173.09	10.18	1.77	4.10E-06	−1.18	0.848
Uridine	243.06	6.85	1.26	3.93E-02	1.18	0.755
Dopamine	152.07	6.41	2.27	7.19E-09	−1.13	0.950
N-isovalerylglycine	158.08	6.89	1.21	6.76E-03	1.11	0.682
Gluconic acid	195.05	12.51	1.05	1.54E-02	−1.10	0.714
Salicylic alcohol	123.05	5.53	1.59	1.54E-05	−1.04	0.848
L-glutamate	146.06	5.47	1.10	8.19E-03	−1.00	0.790
Sebacic acid	201.11	3.94	1.27	3.72E-03	−0.96	0.726
Uracil	111.02	5.00	1.69	1.67E-04	0.96	0.803
Methionine	148.04	9.77	1.72	4.49E-07	−0.94	0.906
Sinapic acid	223.06	5.53	1.66	2.25E-02	−0.93	0.806
L-gulonolactone	177.04	6.25	1.41	1.53E-05	−0.93	0.829
N-acetyl-L-glutamic acid	188.06	12.55	1.45	6.72E-05	−0.92	0.795
Citric acid	191.02	11.29	1.94	3.61E-06	−0.91	0.900
Guanine	150.04	8.40	1.54	6.75E-06	0.90	0.835
3-methyladipic acid	159.07	10.59	1.05	1.32E-02	0.89	0.736
L-cystathione	221.06	14.11	1.36	7.06E-04	−0.89	0.764
Leucine	130.09	7.57	1.46	3.88E-02	−0.85	0.782
Citraconic acid	129.02	12.70	1.42	1.54E-04	−0.85	0.789
Glycyl-L-proline	171.08	12.07	1.67	4.52E-05	−0.84	0.851
SAH	383.11	12.30	1.54	8.69E-05	−0.82	0.823
4-acetamidobutyric acid	144.07	6.70	1.42	1.56E-06	−0.79	0.859
Hydroxyisocaproic acid	131.07	4.26	1.17	1.80E-03	−0.76	0.728
N-acetyl-L-aspartic acid	174.04	12.58	1.15	5.31E-03	−0.69	0.714
Xylitol	151.06	8.83	1.00	3.49E-02	0.68	0.655
6-phosphogluconic acid	194.93	13.81	1.32	2.70E-03	−0.66	0.719
Citramalic acid	147.03	5.51	1.49	4.65E-05	−0.65	0.824
Ascorbic acid	175.02	1.85	1.03	2.95E-02	0.64	0.728
N-acetylneuraminic acid	308.10	12.29	1.09	1.89E-03	−0.62	0.740
Asp-Glu	261.07	14.19	1.20	1.28E-03	−0.60	0.731
Dicrotalic acid	161.04	12.43	1.27	4.06E-03	−0.60	0.730
Isospaglumic acid	303.08	13.70	1.01	1.52E-02	−0.59	0.689
Serine	104.04	12.14	1.09	3.71E-03	0.51	0.736
Cinnamic acid	147.04	9.03	1.05	4.59E-03	−0.41	0.736
3′-O-methylguanosine	296.10	8.30	1.12	3.91E-02	0.37	0.661

^1^mass-to-charge ratio; ^2^retention time; ^3^logarithm of fold change based on two; ^4^area under the curve in receiver operating characteristic curve analysis.

The article "Therapeutic Effects and Metabolic Spectrum of Traditional Chinese Medicine Hengqing II Prescription on Alzheimer's Disease" was published in 2022. Journal: Evid Based Complement Alternat Med.

## Data Availability

The data used to support the findings of this study are included in the article.
